# Establishment of an in vivo rat model for chronic musculoskeletal implant infection

**DOI:** 10.1186/s13018-020-1546-6

**Published:** 2020-01-21

**Authors:** Eivind Witsø, Linh Hoang, Kirsti Løseth, Kåre Bergh

**Affiliations:** 1 Department of Orthopaedic Surgery, St Olav’s University Hospital, Trondheim, Norway; 2 Department of Clinical and Molecular Medicine, Norwegian University of Science and Technology, Trondheim, Norway; 3 Department of Medical Microbiology, St Olav’s University Hospital, Trondheim, Norway

**Keywords:** Experimental, Model, Infection, Chronic, Musculoskeletal

## Abstract

**Background:**

The aim of the study was to establish an experimental chronic musculoskeletal infection model in vivo characterized by (a) a small bacterial inoculum, (b) no general or local signs of infection, (c) several parallels (implants) in each animal and finally (d) a model that is technically easy to perform.

**Methods:**

Bone xenografts with steel plates were implanted intramuscularly in rats. To the xenografts, different inocula of *Staphylococcus aureus* and two strains of *Staphylococcus epidermidis* were added. The animals were observed for different time periods before the removal of the xenografts. The xenografts and steel plates were subjected to quantitative bacterial culture after sonication. Additional steel plates were subjected to scanning electron microscopy (SEM) for visualization of biofilm formation.

**Results:**

Inoculation of bone grafts with *S. aureus* did produce a pyogenic infection in all animals. A chronic infection was established in rats where the bone grafts were inoculated with *S. epidermidis*. A bacterial inoculum of 100 colony-forming units (CFU) of *S. epidermidis* was adequate as a minimum infective dose. During a period of up until 42 days, the animals infected with *S. epidermidis* had no general or local signs of infection. According to the results of the quantitative bacterial culture of sonicate fluid and SEM, a biofilm was developed on all implants.

**Conclusion:**

In the present in vivo model, a very small bacterial inoculum succeeded in establishing a chronic musculoskeletal implant infection where a biofilm was formed on the implants. The experimental model is easy to perform and allows several implants in each animal. The model could be useful for the study of biofilm formation in vivo on different implants and different surfaces.

## Background

A chronic infection is one of the most devastating complications to prosthetic joint surgery. The implant has to be removed, and the final functional result is often much inferior to what the patient would else have expected. These infections are considered to represent biofilm infections [1–3]. Most of the present knowledge of biofilm infections is based on in vitro studies [4]. However, the results of in vitro biofilm studies are not readily reproduced in vivo [5–7], and in vitro biofilm models are not models for the chronic in vivo infection [4]. During the last decades, several experimental models have been used to study the infected orthopaedic implant per se and biofilm formation on the implant in particular [8–22].

In most of the abovementioned models, the foreign body is introduced into or on the tibia or the femur in mouse, rats and rabbits, and there is rarely more than one implant per animal [8–14, 16, 18, 19, 21]. Hence, a large number of animals are needed to achieve many parallels in each experimental group, necessarily implying housing and economic challenges. In some studies, precolonized implants are applied, i.e. the implants are colonized with bacteria in vitro [9, 11, 12, 19, 21]. In a rabbit femur model, Sheehan et al. [14] observed that 10 times more bacteria adhered to the implant when the bacteria were inoculated during the implantation of stainless steel and titanium wires compared to implants precolonized with bacteria.

Many models utilize large bacterial inocula [10, 17], and in some models, the rate of infection of the implants is between 30 and 100% [8, 10, 12, 14]. Finally, many of the models are technically rather demanding and barely possible to perform without being a surgeon.

The purpose of the present work was to establish an experimental model that mimics a chronic orthopaedic implant infection. The experimental model should have the following characteristics: (a) The surgical procedure should be technically easy to perform and allow the use of many parallels in relatively few animals. (b) A small bacterial inoculum should result in a chronic infection on all implants. Finally, (c) the infection established should have the characteristics of a chronic orthopaedic infection with no local or general signs of a purulent infection.

## Methods

### An overview of the design of the study

The Norwegian Council for Animal Experimentation approved the study (FOTS nr. 3854, 3987 and 4402). Rats were operated with intramuscular implantation of two bone grafts each containing two steel plates (Fig. 1). The bone grafts were seeded with strains of either *Staphylococcus aureus* (American Type Culture Collection (ATCC) 25923), *S. epidermidis* (ATCC 35984) and *S. epidermidis* (ATCC 12228) [21–23].

**Fig. 1:** **a**, **b** Xenograft and implants used for establishing a chronic infection model. Steel plates were impacted in both ends of a corticospongious xenograft (lamb costae)

The extent of infection was evaluated by clinical observation of the animals and post mortem culture of muscle and spleen biopsies and quantitative culture of sonicated bone grafts. The degree of biofilm formation on steel plates was evaluated by sonication of the steel plates, followed by quantitative culture of the sonicate fluid and scanning electron microscopy (SEM) of the plates.

Three experiments were conducted:

1. Ten rats were operated with five rats in each experimental group. The bone grafts were inoculated with a 10-μl suspension containing 10^4^ colony-forming units (CFU) of *S. aureus* (ATCC 25923) and *S. epidermidis* (ATCC 35984), respectively. After 20 days, the bone grafts with their content were removed and further processed. Biopsies from the spleen and muscle surrounding the implants were collected for culture.
2. Twenty rats were operated, 10 rats in each experimental group. The bone grafts were inoculated with a 10-μl suspension of *S. aureus* (ATCC 25923) and *S. epidermidis* (ATCC 35984), respectively. In each experimental group, the bone grafts were contaminated with 10^4^, 10^3^ and 10^2^ CFU in each subgroup of three rats, respectively. After 42 days, the bone grafts with their content were removed and further processed. Biopsies from the muscle were collected for culture.
3. Ten rats were operated, five rats in each experimental group. The bone grafts were inoculated with a 10-μl suspension of 10^2^ CFU of *S. epidermidis* (ATCC 35984) and *S. epidermidis* (ATCC 12228), respectively. After 26 days, the bone grafts were removed and further processed. Biopsies from the muscle were collected for culture.

In each experimental group, one rat acted as a negative in vivo control.

### Bacterial strains

Overnight cultures of *S. aureus* (ATCC 25923) and *S. epidermidis* (ATCC 35984 and ATCC 12228) were dissolved in 5% glucose broth and incubated in order to obtain log-phase growth. Ten-microliter aliquots of bacterial solution were serially diluted and seeded at regular time intervals after spectrometrical measurements enabling a standard curve for bacterial concentrations. This procedure allowed us to make the following 10-μl inoculate applied in the respective experiments: 10^4^, 10^3^ and 10^2^ CFU of ATCC 25923 and ATCC 35984 and 10^2^ CFU of ATCC 12228.

The respective bacterial solutions were kept on ice and brought to the Department of Comparative Medicine Core facility. Samples in duplicate from the bacterial solutions were seeded on blood agar plate at regular intervals during the operations to confirm the inoculum employed.

All seeded agars were incubated overnight at 37 °C and enumerated in by using aCOLyte Colony Counter (Synbiosis, Cambridge, UK). In all experiments, representative colonies of bacteria harvested from infected animals were processed for pulsed-field gel electrophoresis using BIO-RAD CHEF MAPPER™ XA and compared with ATCC 25923, ATCC 35984 and ATCC 12228, respectively.

### The implant

One hundred sixty steel plates (AISI 316-L, Scandinavian Customized Prosthesis®), 5 × 5 × 1 mm, Ra 0.20 (0.12–0.31) μm, were sonicated (40 kHz, 200 W, BactoSonic®, Bandelin GmbH, Berlin) in sterile water for 2 × 15 min before sterilization by autoclaving.

### The bone grafts

Lamb costa from Norwegian white sheep was obtained from the slaughterhouse (Nortura Malvik®, 7550 Hommelvik, Norway). The lambs had not been given any medication before they were killed by electricity. From the mid part of costae, 80 pieces of corticocancellous bone grafts were cut manually with a saw. With an electric sanding machine, the periost was removed and sharp corners were rounded. The grafts were 15.3 (14.5–16.5) mm in length and 11.9 (10.5–13.0) mm in breadth, and they weighted 1.16 (1.00–1.27) g. A groove was made with a surgical knife in each end of the bone graft before a steel plate was gently inserted into each end of the graft with a forceps until the outer end of the steel plates were even with the cortical bone. At the mid part of the graft, a small hole was made into the bone marrow with a 1.9-mm drill (Fig. 1). The bone graft with the implant was then sterilized.

### The operation

All operations were performed in a laminar air flow cabinet under standard operation theatre conditions. Forty male albino, outbred Wistar rats (HanTac:WH, Taconic, Denmark), 13 weeks old [12–14] and 360 (312–413) g, were operated. In all experiments, the operation field was shaved and washed with 70% ethanol. The animals were placed on sterile drapes, and their bodies were covered with sterile sheets, with a hole exposing the operation field. In all operations, the rats were given general sedation, and if necessary, buprenorphin as postoperative pain treatment. At the end of the experiment, the rats were killed with an intracardial injection of pentobarbital.

Briefly, a 4-cm-long incision was made in the midline at the proximal part of the back, and a subfascial/intramuscular cavity was made with a scissor on each side of the midline (right = A, left = B). Ten microliters of the respective bacteria solution was injected into the hole on the mid part of the bone graft 3 s before the bone grafts with the steel plates were implanted in each subfascial/intramuscular cavity. In animals that acted as negative in vivo controls, the bone grafts were implanted directly into the cavities without any bacterial seeding. The skin was closed with a continuous locking madras suture. All animals were operated separately, with new dressing and instruments for each animal. During the first 24 h postoperatively, the animals were kept in separate cages and thereafter three and three in each cage. The animals were housed in a 12-h-night-day cycle environment. They were allowed free movement, standard food (rat and mouse diet “BKOO1E) and water ad libitum. The animals were weighed on the day of surgery and at weekly intervals throughout the study period. They were inspected daily for any complications, in particular signs of purulent wound secretion.

At the end of the experiment, a 5 × 5 × 5-mm biopsy was first taken from the spleen by a laparotomy (experiment I). The old scar at the back of the animal was then opened, and any possible signs of local infection were noted. Two 5 × 5 × 5 mm biopsies were harvested from the muscle surrounding the bone grafts. The bone grafts were then removed, first graft A and then graft B. By applying a gentle pressure by forceps over the mid part of the graft, the graft would split longitudinally and then the graft could be opened like a book. One of the two steel plates from bone graft A was immediately put in fixation solution for SEM. Next, the bone grafts with its content were separately put into sterile plastic containers and were immediately placed on ice for further processing.

The duration of the two surgical procedures in each animal was approximately 10 and 7 min, respectively.

### Postoperative processing of spleen biopsies, muscle biopsies, bone grafts and steel plates

All specimens were kept on ice and brought to the laboratory for immediately processing.

The spleen biopsies were grounded in a mortar with 1 ml of sterile saline, after which 50 μl of the suspension was seeded onto blood agar plate. The muscle biopsies were grounded with 3 ml of sterile saline, the suspension was serially diluted and 10 μl was seeded onto blood agar plate. While still on ice, each steel plate was removed from the bone grafts with a pincer. In a sterile plastic tube with 3 ml saline, each steel plate was gently stirred (600 rpm) for 10 s. This washing procedure was repeated twice (three times in experiment II), and the steel plate was transferred each time with a new sterile pincer. After the last washing procedure, the plate was transferred to a sterile glass tube with 3 ml sterile saline for removal of biofilm [24]. Briefly, the glass tube with its content was vortex mixed at 2400 rpm for 30 s, followed by sonication (40 kHz, 200 W, BactoSonic®, Bandelin GmbH, Berlin) for 5 min, and then a second vortex mixing at 2400 rpm for 30 s. Ten microliters of the sonicate fluid was serially diluted and seeded onto blood agar plate. After completion of sonication, the second steel plate from bone graft A was put into a fixation solution for SEM. Finally, the bone grafts were vortex mixed and sonicated in 6 ml of sterile saline according to the same procedure as the steel plates (preliminary studies had shown that this procedure yielded an equivalent amount of bacteria as if the bone grafts had been grounded in a mortar). From this sonicate fluid, 10 μl was serially diluted and seeded onto a blood agar plate.

From the three animals that acted as negative in vivo control, one plate from each of the bone grafts was processed directly for SEM, while the other plates were sonicated. After sonication, aliquots of sonicate fluid were seeded onto a blood agar plate. Sonicated plates from negative in vivo control animals were processed for SEM.

### Scanning electron microscopy (SEM) of steel plates

For SEM, the steel plates were briefly rinsed with 0.1 M Hepes buffer (Sigma-Aldrich) at pH 7.2, then fixed in 2.5% glutaraldehyde (Chemi-Teknik AS), 2% paraformaldehyde (VWR, Part of Avantor) and 0.075% Ruthenium Red (Sigma-Aldrich) in 0.1 M Hepes buffer for 4 h at room temperature. Afterwards, the specimens were rinsed in 0.1 M Hepes buffer and then dehydrated through a graded series of ethanol (Antibac AS), (10%, 25%, 50%, 70%), and 90%] for 7 min each and then 3 times in 100% ethanol for 10 min each. After dehydration, the specimens were dried using a chemical hexamethyldisilazane (HMDS) (Sigma-Aldrich), first exchange with 50% solution of HMDS diluted with 100% ethanol for 20 min, then three exchanges with 100% HMDS for 20 min each. Finally, HMDS were removed and the specimens were allowed to air-dry in a fume hood overnight. Dried samples were mounted on stubs using double-sided conductive adhesive carbon tape (both from Chemi-Teknik AS). Specimens were then coated with a 30-nm-thick layer of gold/palladium (Au/Pd) using a sputter coater (polaron) (2.5 kV, 20 mA, 3 min). Specimens were examined with a JSM 6480 (JEOL) scanning electron microscope with digital imaging capabilities. The secondary electron images were collected at an acceleration voltage of 20 kV and digitalized as TIFF computer files.

### Presentation of data

Data are presented as either mean (total range) or mean ± 1 standard deviation (SD).

## Results

### Animals infected with *S. aureus* (ATCC 25923)

In brief, inoculating the bone grafts with *S. aureus* resulted in an acute postoperative infection, and none of the animals (*n* = 13) infected with *S. aureus* developed a chronic infection. All animals had macroscopic signs of a purulent infection in the subcutaneous and muscle tissue. In experiment I, the total number of CFU in the eight bone grafts contaminated with *S. aureus* was 46 (± 32)·10^7^. One steel plate was lost during processing, leaving 11 steel plates for sonication. The CFU/millilitre in sonicate fluid was 65 (± 40)·10^4^. Plates prepared for SEM showed bacterial colonization on all plates.

None of the rats infected with *S. aureus* fulfilled experiment II: after 24 days, 4/9 rats had severe purulent wound infections and the animals were sacrificed. In the other 5/9 rats, the bone grafts had already been spontaneously expelled.

### Animals infected with *S. epidermidis* (ATCC 35984 and ATCC 12228)

Of the 25 animals, one rat died postoperatively due to respiratory depression. In one animal, the bone grafts and the implants were infected with a *S. aureus* contaminant (different from ATCC 25923). In the rest of the infected animals (*n* = 19), the causative microbe was identified as ATCC 35984 and ATCC 12228, respectively. All animals, including controls (*n* = 23), were healthy and gained weight, and cultures of biopsies from the spleen were negative.

In the 19 infected animals, there were no macroscopic signs of infection of the skin in the subcutaneous or subfascial tissue. All bone grafts remained positioned intramuscularly. In five animals, the bone grafts were surrounded by a pseudocapsule filled with sanguinolent fluid. ATCC 35984 and ATCC 12228 were cultured in respective biopsies taken from the muscle adjacent to the contaminated bone grafts. The total number of CFU in bone grafts at the right side of the animal (graft A) and the left side (graft B) was similar (data not shown). Irrespective of the bacterial inoculum, the length of the infectious period and the bacterial species (*S. epidermidis* ATCC 35984 and *S. epidermidis* ATCC 12228), the total number of CFU in bone grafts were about 10^7^ and bacterial growth in sonication fluid was about 10^3^ CFU/ml (Tables 1 and 2). Examination with SEM showed bacterial growth, individually and in colonies, on all plates contaminated with *S. epidermidis* (Fig. 2a–c).

**Table 1:** Steel implants infected with *S. epidermidis* ATCC 35984 in an in vivo rat model

Inoculum (CFU)	0.7 (0.7–0.8) 10^4^	1.1 (1.1–1.1) 10^4^	0.9 (0.7–1.1) 10^3^	1.4 (1.3–1.4) 10^2^
Time period (days)	20	42	42	42
Rats (*n*)	4	2^a^	3	2^a^
Bone grafts (*n*)	8	4	6	4
Steel plates (*n*)^b^	12	6	9	6
Bacterial growth in bone grafts (total CFU)	110 (± 50)·10^5^	69 (± 41)·10^5^	96 (± 65)·10^5^	170 (± 36)·10^5^
Bacterial growth in sonicate fluid (CFU/ml)	217 (± 122)·10^2^	31 (± 22)·10^2^	68 (± 112) 10^2^	32 (± 21) 10^2^

The total number of CFU of *S. epidermidis* ATCC 35984 are listed as a result of different time periods for infection and different inoculum size (experiments I and II). The number of CFU recovered from bone grafts and sonicate fluid are presented as mean (± 1 SD).

^a^One rat died postoperatively. In one rat, the bone grafts were contaminated

^b^From each animal, one steel plate was processed for SEM and three steel plates were sonicated

**Table 2:** Recovery of bacteria from rats inoculated with a small inoculum of two *S. epidermidis* strains

	ATCC 35984	ATCC 12228
Inoculum (CFU)	1.02 (0.80–1.12)·10^2^	0.92 (0.87–1.04)·10^2^
Rats (*n*)	4	4
Bone grafts (*n*)	8	8
Steel plates (*n*)^a^	12	12
Bacterial growth in bone grafts (total CFU)	341 (± 266)·10^5^	109 (± 79)·10^5^
Bacterial growth in sonicate fluid (CFU/ml)	159 (± 100)·10^2^	113 (± 94)·10^2^

^a^From each animal, one steel plate was processed for SEM and three steel plates were sonicated

The number of CFU in bone grafts and sonicate fluid are presented as mean (± 1 SD)

**Fig. 2:** **a**–**c** Scanning electron micrograph showing bacterial growth with biofilm in small colonies on steel plates (*S. epidermidis*, ATCC 35984)

In control animals, no bacterial growth was recorded in the spleen tissue, muscle tissue, bone graft or sonicate fluid. No bacteria were observed on steel plates prepared for SEM.

## Discussion

We here present a new experimental model for the study of chronic implant infections in the musculoskeletal system. We found that a bone xenograft with implants contaminated with a very low inoculum of *S. epidermidis* in this in vivo model resulted in a chronic implant infection.

Numerous models for in vivo studies of skeletal staphylococci implant infections have been presented during the last 50 years [22, 25]. In vivo studies are justified due to the interaction between the host, the bacteria and the implant, which cannot be studied in vitro [26]. Furthermore, clinical trials on osteomyelitis are difficult to conduct due to a large variability of the disease, a low incidence in most countries, a heterogeneous population and a broad range of causative microbes [22, 25].

The strength of the present study is that a very small inoculum (100 CFU) of *S. epidermidis* was capable of establishing a chronic infection, and a biofilm was formed on all implants. This is probably more comparable to the clinical situation of preoperative contamination of devices as opposed to the massive infectious doses often employed in many experimental in vivo models. Even after 6 weeks, none of the animals infected with *S. epidermidis* had general or local signs of an infection, and the animals had a normal gain in body weight. The model allowed several implants (parallels) in each animal, thus reducing the number of experimental animals needed. In the present study, a total of two xenografts and four implants were studied in each animal, but the number of grafts (implants) could easily have been doubled. The surgical technique applied in the present model is easy to perform. After training and supervision, operation of the animals can be performed by personnel not necessarily possessing complete surgical skills. Finally, in the present model, the risk of bacterial contamination from the fur and skin of the animal was negligible. Sonication of bone grafts and steel plates in the present study was performed according to standard procedure [27]. Bacterial growth in sonicate fluid has been considered a proof of the presence of biofilm in both in vitro and clinical studies [27–30]. In the present study, SEM was employed to visualize the presence of bacterial adherence on steel plates. This is a qualitative evaluation which has been used in both in vitro and clinical studies [31, 32]. In a pilot study, we tried to quantify the number of bacterial colonies (i.e. more than five bacteria in a cluster). At a magnification of × 2000 we scanned about 7% of the total area of the plate. This method allowed us to quantify the total number of bacterial colonies in plates subjected to the same experimental setup, and we found that parallels had a similar number of bacterial colonies (data not shown). This procedure was extremely time-consuming. But at least it was possible to quantify the number of bacterial colonies on the plate, as opposed to what would have been feasible on a curved surface, as for example the surface of pins. In the present study, neither bacterial culture of sonicate fluid nor SEM was employed quantitatively, but as a means to study if even an extremely small bacterial inoculum could create a chronic biofilm infection.

The finding of a low-virulent bacterium as *S. epidermidis* resulting in a chronic infection is in accordance with clinical observations [33]. In the present study, we used a biofilm-forming *S. epidermidis* (ATCC 35984) and a non-biofilm-forming *S. epidermidis* (ATCC 12228) [23, 34]. As observed in other studies, the differences in biofilm-forming abilities were not reproduced in vivo [6, 7]. To our best knowledge, this observation has not been further addressed in specific experimental models of orthopaedic implant infections.

A weakness of the present study includes that we did not manage to create a chronic infection when the xenografts were contaminated with *S. aureus.* Other authors have succeeded in creating a chronic infection in rat femora when a foreign body introduced intramedullary (pin or wire) was contaminated with *S. aureus* [22]. In our model, *S. aureus* resulted in an acute suppurative infection, probably due to the avascular status of the xenograft and the virulence of the organism. We do not know to what degree the use of a xenograft will influence on the applicability of the model. However, the present model is first and foremost a model for studying implant infections, and not a model for studying osteomyelitis.

The limitations of the present study were that only one bacterial species (i.e. staphylococci) and one type of implant (i.e. steel) were studied. Inoculation with other low-virulent bacteria, as for example *Cutibacterium acnes*, would possibly also result in a chronic infection, but this has yet to be shown. We could have used other imaging techniques, both to make a qualitative and quantitative evaluation of the presence of a biofilm. Confocal laser scanning microscopy has been employed to study the biofilm per se in vivo [21, 31]. A quantitative evaluation of biofilm formation has been studied with different fluorescence techniques and with different degree of success [21, 35]. Jørgensen et al. [21] employed a mouse model where precolonized pins were inserted into mouse tibia. Bioluminescent *S. aureus* allowed bioluminescent imaging. However, bioluminescence activity decreased during the study period although the bacterial load was the same. This phenomenon was explained by precolonization of the implants and emphasizes that culture of sonication fluid was the most reliable quantitative method. Finally, the results observed in this model do only relate to rats. Rats are known to have a strong immune system [22], and other results could have been observed if for example rabbits had been used.

## Conclusions

The present model is primarily a model for the study of biofilm formation on implants in vivo*.* A very small and clinically relevant bacterial inoculum creates a low virulent chronic implant infection with no macroscopic sign of infection. The model could be employed when the effect of local antibiotics or surface modification of the implant is the subject of interest. The present in vivo model could possibly also be used to study the effect of per oral or parenteral antibiotic treatment in cases of musculoskeletal and foreign body infections, but this has to be explored.

## Data Availability

All data generated and analyzed during this study are included in this published article.

## Abbreviations

ATCC: American Type Culture Collection
CFU: Colony-forming units
SEM: Scanning electron microscopy
